# The Investigation of the Application Value of Musculoskeletal Ultrasound in the Diagnosis and Conservative Treatment of Knee Osteoarthritis

**DOI:** 10.1155/2022/9660067

**Published:** 2022-08-16

**Authors:** Yan Pan, Liying Wang, Lingling Zhou

**Affiliations:** The Affiliated Yantai Yuhuangding Hospital of Qingdao University, China

## Abstract

**Objective:**

To explore the application value of musculoskeletal ultrasound in the diagnosis and conservative treatment of knee osteoarthritis.

**Methods:**

Patients with knee osteoarthritis who were treated in our hospital from January 1, 2020 to August 31, 2021 were selected as the research subjects. The subjects underwent musculoskeletal ultrasonography to record the thickness of the lateral femoral malleolus cartilage, the thickness of the medial femoral malleolus cartilage, the depth of the suprapatellar bursa effusion, and the thickness of the suprapatellar bursa synovium. All patients in the study group received acupuncture treatment after musculoskeletal ultrasonography, and musculoskeletal ultrasonography was performed again after 2 weeks of treatment. The differences in musculoskeletal ultrasound-related parameters were compared between the two groups.

**Results:**

The thickness of the lateral femoral malleolus cartilage and medial femoral malleolus cartilage in the study group was significantly smaller than those in the control group. The depth of the effusion in the suprapatellar bursa and the thickness of the synovial membrane in the suprapatellar bursa were significantly greater than those in the control group. Ultrasonography showed no significant difference in abnormal status compared with arthroscopy, and musculoskeletal ultrasonography revealed knee osteoarthritis, such as cruciate ligament injury, joint effusion, synovial hyperplasia, meniscus injury, and patellar ligament injury. The cartilage thickness of the lateral femoral malleolus and medial malleolus of femur after treatment were significantly greater than those before treatment. The depth of the deep suprapatellar bursa effusion and the thickness of the suprapatellar bursa synovium were significantly smaller than those before treatment.

**Conclusion:**

Musculoskeletal ultrasound has high diagnostic value in knee osteoarthritis. It can detect the lesion as soon as possible and can be used to evaluate the effect of conservative treatment, so as to provide reference basis for clinical formulation or adjustment of further intervention plan.

## 1. Introduction

Knee osteoarthritis is a multiple chronic degenerative joint disease in middle-aged and elderly people. It is mainly caused by the degradation of extracellular matrix, chondrocytes, and subchondral bone under the joint action of many biological and mechanical factors, and the normal coupling of synthesis is abnormal. It can be secondary to narrow joint space, joint capsule contracture, and synovitis, resulting in different degrees of joint dysfunction and pain. It poses a great threat to the physical and mental health and quality of life of patients [1–3]. Therefore, early diagnosis of knee osteoarthritis and accurate evaluation of disease treatment are of great significance to guide clinical targeted intervention.

CT and MRI are important imaging diagnostic techniques in clinic. They have a certain diagnostic value in knee osteoarthritis, but it is difficult to present information such as tissue hardness, resulting in limitations in their clinical application [4, 5]. Ultrasound is also a common clinical diagnostic method. It has the advantages of simple operation, low inspection cost, and noninvasive and can effectively present the situation of joint-related tissues [6, 7].

In this study, patients with knee osteoarthritis who were treated in our hospital were used as the research objects, and a control group was established to conduct a controlled study to clarify the application value of musculoskeletal ultrasound in the diagnosis and conservative treatment of knee osteoarthritis.

## 2. Methods

### 2.1. Patients

Patients with knee osteoarthritis who were treated in our hospital were used as the research objects. The inclusion criteria were as follows: (1) the research group met the diagnostic criteria for knee osteoarthritis [8], (2) the patients were able to cooperate in completing the investigation and research, (3) informed consent to this study and signed the paper consent form voluntarily, and (4) age < 80 years old. The exclusion criteria were as follows: (1) patients with obvious bone hyperplasia, (2) patients with joint trauma, (3) arthritis caused by other factors, such as chloasma and syphilitic neuropathy, (4) 3 months before the study, (5) mentally ill patients, (6) lactating/pregnant women, and (7) body mass index (BMI) > 30 kg/m^2^.

### 2.2. Diagnostic Method

All subjects were examined by musculoskeletal ultrasound. The equipment was Philips EPIQ 5 color Doppler ultrasound diagnostic instrument, and the high-frequency probe was adopted. The probe frequency was set to 5 ~ 13 MHz. The patient was guided to take the flat lying or sitting position, bend both knees, and fully expose the knee cartilage. The probe is applied with conductive couplant, and the abnormal part is identified by dynamic scanning of the ultrasonic probe along the long axis of the muscle, and the probe is rotated 90° to scan and scan the synovial sac, ligament, tendon, and muscle and measure the depth and extent of the effusion. The thickness of the femoral lateral malleolus cartilage, femoral medial malleolus cartilage, and suprapatellar capsule synovium was recorded.

### 2.3. Treatment Method

Patients in the study group received little needle knife treatment after musculoskeletal ultrasound examination. The experience acupoints and tenderness points were selected as the feeding point, patients were guided to take the flat lying position, 2.5 ml lidocaine (2%) was injected layer by layer into the skin and periosteum at the feeding point for local anesthesia, Hanzhang needle knife (No. 4) was used to pierce along the pinhole and cut and peel off the nodules and cords, and the needle knife was withdrawal after loosening, the pinhole was compressed with sterile cotton ball, and the pinhole was pasted with dressing. Popliteal tenderness points and experience points were treated with the same method. After 2 weeks of treatment, musculoskeletal ultrasound examination was performed again. The thickness of the femoral lateral malleolus cartilage, femoral medial malleolus cartilage, the depth of the suprapatellar capsule effusion, and the thickness of the suprapatellar capsule synovium were measured.

### 2.4. Observation Indicators

Musculoskeletal ultrasound parameters in the two groups were counted and compared, including the thickness of the femoral lateral malleolus cartilage and femoral medial malleolus cartilage, the depth of the suprapatellar capsule effusion, and the thickness of the suprapatellar capsule synovium. Arthroscopic diagnosis was taken as the reference, and diagnosis of knee osteoarthritis by musculoskeletal ultrasound was counted and analyzed. Musculoskeletal ultrasonic parameters before and after treatment in the study group were counted and analyzed (the thickness of the femoral lateral malleolus cartilage and femoral medial malleolus cartilage, the depth of the suprapatellar capsule effusion, and the thickness of the suprapatellar capsule synovium).

### 2.5. Statistical Analysis

The SPSS version 22.0 (IBM SPSS statistics, USA) was used for data analysis. Measurement data was expressed as mean ± *s*; *t*-test was used for data analysis. The two-sided *P* < 0.05 indicated the difference was statistically significant.

## 3. Results

### 3.1. Baseline Data

We enrolled 93 patients in this study, but 8 patients failed to meet the inclusion criteria were excluded. A total of 85 patients with knee osteoarthritis from January 1, 2020 to August 31, 2021 in our hospital were selected as the study group, and another 85 healthy cases at the same period were selected as the control group. There were 47 males and 38 females in the study group. The age ranged from 37 to 76 years, with an average of 56.64 ± 14.07 years; disease grade: 10 cases of grade 0, 17 cases of grade I, 19 cases of grade II, 26 cases of grade III and 13 cases of grade IV; The course of disease ranged from 1.5 to 12.5 years, with an average of 7.11 ± 3.69 years. There were 49 males and 36 females in the control group. The age ranged from 35 to 79 years, with an average of 57.18 ± 12.95 years. The clinical data of the two groups were balanced and comparable (*P* > 0.05), and this study was approved by the ethics committee of our hospital.

### 3.2. Comparison of Musculoskeletal Ultrasound Parameters between the Two Groups

The thickness of the femoral lateral malleolus cartilage (1.61 ± 0.49 mm) and femoral medial malleolus cartilage (1.39 ± 0.24 mm) in the study group was less than those in the control group (femoral lateral malleolus cartilage thickness (1.95 ± 0.50 mm), femoral medial malleolus cartilage thickness (1.96 ± 0.44 mm)); the depth of the suprapatellar capsule effusion (11.45 ± 2.59 mm) and the thickness of the suprapatellar capsule synovium (3.41 ± 1.59 mm) were greater than those in the control group (suprapatellar capsule effusion depth (2.42 ± 0.89 mm), synovial thickness of the suprapatellar capsule (0.95 ± 0.39 mm)); the difference was statistically significant (*P* < 0.05), as shown in Table 1.

### 3.3. Comparison of Diagnosis of Knee Osteoarthritis by Musculoskeletal Ultrasound between the Two Groups

There was no significant difference in the abnormal status of ultrasonic examination of knee osteoarthritis by musculoskeletal ultrasound, such as cruciate ligament injury (100.00%), joint effusion (97.01%), synovial hyperplasia (94.92%), meniscus lesions (85.71%), and patellar ligament lesions (100.00%) compared with arthroscopy (100.00%, 100.00%, 98.31%, 100.00%, and 100.00%) (*P* > 0.05), as shown in Table 2.

### 3.4. Comparison of Musculoskeletal Ultrasonic Parameters before and after Treatment in the Study Group

After treatment, the thickness of the femoral lateral malleolus cartilage was 1.87 ± 0.46 mm and the thickness of the femoral medial malleolus cartilage was 1.84 ± 0.37 mm, which was greater than that before treatment (the thickness of the femoral lateral malleolus cartilage was 1.61 ± 0.49 mm and the thickness of the femoral medial malleolus cartilage was 1.39 ± 0.24 mm); the depth of the suprapatellar capsule effusion was 4.65 ± 1.13 mm and the thickness of the suprapatellar capsule synovium was 1.23 ± 0.46 mm, which was less than that before treatment (the depth of the suprapatellar capsule effusion was 11.45 ± 2.59 mm, and the thickness of the suprapatellar capsule synovium was 3.41 ± 1.59 mm); the difference was statistically significant (*P* < 0.05), as shown in table 3.

## 4. Discussion

Knee osteoarthritis is a clinical multiple disease. Its pathogenesis lies in the scar adhesion caused by the injury of soft tissue around the knee joint, which leads to the long-term contracture and degeneration of soft tissue. It can cause the loss of physiological function of the knee joint and abnormal biomechanical balance, which has a great impact on the daily activities and life of patients [9, 10]. At the same time, timely and effective intervention for patients with early knee osteoarthritis can alleviate the clinical symptoms, restore joint function, and inhibit the progress of the disease, which is of great significance to improve the activity ability and quality of life of patients [11, 12]. In recent years, with the aging of population, the incidence rate of knee osteoarthritis has been increasing. It has become an important cause of the loss of working ability or exercise ability of the middle-aged and elderly [13]. Therefore, how to accurately diagnose and evaluate knee osteoarthritis is still a hot spot in study.

At present, there are many clinical diagnostic measures for knee osteoarthritis, of which X-ray film and MRI are commonly used. X-ray film is widely used and cheap, but it can only clearly show the bone structure. As a result, most patients with knee osteoarthritis diagnosed by X-ray film are in the middle and late stage, not only cartilage injury but also joint deformity and hyperosteogeny, so they need total knee arthroplasty [14, 15]. MRI is not suitable for early screening of knee osteoarthritis because of its low specificity and high cost, although it has a better display effect of the bone marrow edema, joint ligament, and synovium. Musculoskeletal ultrasound is a diagnostic technique applied in the diagnosis and evaluation of bone and joint diseases in recent years. It has unique diagnostic value in joint effusion, bone invasion, synovial hypertrophy and hyperplasia, blood flow, and cartilage injury [16, 17]. Relevant studies have shown that patients with knee osteoarthritis can have thinning of the cartilage layer and reduction of the cartilage in the early stage. Such signs can be detected by ultrasound, and there is a positive correlation between the degree of cartilage degeneration and the duration of knee osteoarthritis [18, 19]. The results showed that the thickness of the femoral lateral malleolus cartilage and femoral medial malleolus cartilage in the study group was less than those in the control group, the depth of the suprapatellar capsule effusion and the thickness of the suprapatellar capsule synovium were greater than those in the control group (*P* < 0.05), and there was no significant difference between musculoskeletal ultrasound and arthroscopy in the detection rate of abnormal ultrasonic examination of knee osteoarthritis (*P* > 0.05), indicating that musculoskeletal ultrasound has high diagnostic value in knee osteoarthritis and can detect the lesions. The reason is that musculoskeletal ultrasound can effectively reflect the lesions of the articular cartilage and the proliferation of blood vessels around the articular surface, so as to improve the diagnostic efficiency.

In addition, musculoskeletal ultrasound was used to examine and evaluate the relevant signs of patients with knee osteoarthritis. The results showed that the thickness of the femoral lateral malleolus cartilage and femoral medial malleolus cartilage after treatment was greater than those before treatment, and the depth of suprapatellar capsule effusion and the thickness of the suprapatellar capsule synovium were less than those before treatment (*P* < 0.05), suggesting that musculoskeletal ultrasound can effectively determine the changeable situation of joint effusion and the thickness of the articular cartilage. This is mainly because the operation of musculoskeletal ultrasound is simple, which can show the characteristics of the meniscus, synovium, and other anatomical structures, so as to dynamically observe the muscles and tendons, clearly identify the superficial organs, and accurately reflect the state of peripheral nerves and blood vessels, especially in the diagnosis of soft tissue diseases [20]. However, it should also be noted in clinical practice that musculoskeletal ultrasound has its own limitations in the diagnosis and evaluation of knee osteoarthritis, that is, some patients with knee osteoarthritis have severe limited joint flexion, joint space disappears or is narrow, and the sound velocity is difficult to pass through the joint cavity, which can affect the presentation effect of the cartilage tissue of the femoral head and tibial plateau, and the inspection and evaluation results will be affected by the operator's technology and subjective experience to a certain extent [21].

In summary, musculoskeletal ultrasound has a high diagnostic value in knee osteoarthritis. It can detect the lesion as soon as possible and can be used to evaluate the effect of conservative treatment, so as to provide reference basis for clinical formulation or adjustment of further intervention plan. However, this study did not compare the ultrasound findings of patients with knee osteoarthritis of different severity before and after treatment, and it was a small sample study, so further clinical research is still needed.

## Figures and Tables

**Table 1:** Comparison of musculoskeletal ultrasound parameters between the two groups.

Groups	Cases	Thickness of femoral lateral malleolus cartilage	Thickness of femoral medial malleolus cartilage	Depth of suprapatellar capsule effusion	Thickness of suprapatellar capsule synovium
The study group	85	1.61 ± 0.49	1.39 ± 0.24	11.45 ± 2.59	3.41 ± 1.59
The control group	85	1.95 ± 0.50	1.96 ± 0.44	2.42 ± 0.89	0.95 ± 0.39
*t* value		4.478	10.485	30.399	13.854
*P* value		*P* ≤ 0.01	*P* ≤ 0.01	*P* ≤ 0.01	*P* ≤ 0.01

**Table 2:** Comparison of diagnosis of knee osteoarthritis by musculoskeletal ultrasound between the two groups.

Groups	Cruciate ligament injury (*n* = 8)	Joint effusion (*n* = 67)	Synovial hyperplasia (*n* = 59)	Meniscus lesions (*n* = 7)	Patellar ligament lesions (*n* = 11)
Musculoskeletal ultrasound	8 (100.00)	65 (97.01)	56 (94.92)	6 (85.71)	11 (100.00)
Arthroscope	8 (100.00)	67 (100.00)	58 (98.31)	7 (100.00)	11 (100.00)
*χ* ^2^ value	0.000	0.508	0.259	0.000	0.000
*P* value	1.000	0.476	0.611	1.000	1.000

**Table 3:** Comparison of musculoskeletal ultrasonic parameters before and after treatment in the study group.

Group	Cases	Thickness of femoral lateral malleolus cartilage	Thickness of femoral medial malleolus cartilage	Depth of suprapatellar capsule effusion	Thickness of suprapatellar capsule synovium
Before treatment	85	1.61 ± 0.49	1.39 ± 0.24	11.45 ± 2.59	3.41 ± 1.59
After treatment	85	1.87 ± 0.46	1.84 ± 0.37	4.65 ± 1.13	1.23 ± 0.46
*t* value		3.567	9.407	22.186	12.143
*P* value		*P* ≤ 0.01	*P* ≤ 0.01	*P* ≤ 0.01	*P* ≤ 0.01

## Data Availability

Data will be available upon request.

## References

[1] Li X. F., Sun Y. L., Zhou Z. L. (2019). Mitigation of articular cartilage degeneration and subchondral bone sclerosis in osteoarthritis progression using low-intensity ultrasound stimulation. *Ultrasound in Medicine & Biology*.

[2] Li S. H., Yang M., Tang L., Zhou Y. (2021). The synergistic effects of applying low-level laser therapy plus ultrasound on pain and muscle function in patients with knee osteoarthritis: a protocol of a randomized double-blind study. *Medicine (Baltimore)*.

[3] Liu J., Xiu Z. B., Lin Q. X., Lu L. M., Guo Z. X., Gong Y. R. (2021). Ultrasound anatomy and needle-knife insertion approach of common tendon lesions in knee osteoarthritis based on meridian sinew theory. *Zhongguo Zhen jiu= Chinese Acupuncture & Moxibustion*.

[4] Xiang X., Liu H., Wang L. Y. (2020). Ultrasound combined with SDF-1*α* chemotactic microbubbles promotes stem cell homing in an osteoarthritis model. *Journal of Cellular and Molecular Medicine*.

[5] Ozgonenel L., Okur S. C., Dogan Y. P., Çaglar N. S. (2018). Effectiveness of therapeutic ultrasound on clinical parameters and ultrasonographic cartilage thickness in knee osteoarthritis: a double-blind trial. *Ultrasound*.

[6] Thomas M., Petterson S., Plancher K. (2020). Sustained acoustic medicine as a non-surgical and non-opioid knee osteoarthritis treatment option: a health economic cost-effectiveness analysis for symptom management. *Journal of Orthopaedic Surgery and Research*.

[7] Luo Q. L., Ji S. H., Li Z. M., Huang T., Fan S., Xi Q. (2019). Effects of ultrasound therapy on the synovial fluid proteome in a rabbit surgery-induced model of knee osteoarthritis. *Biomed Eng Online*.

[8] Bannuru R. R., Osani M. C., Vaysbro E. E. (2019). OARSI guidelines for the non-surgical management of knee, hip, and polyarticular osteoarthritis. *Osteoarthritis and Cartilage*.

[9] Zhou X. Y., Zhang X. X., Yu G. Y. (2018). Effects of low-intensity pulsed ultrasound on knee osteoarthritis: a meta- analysis of randomized clinical trials. *BioMed Research International*.

[10] David O., Klyve D., Ortiz R., Best T. M. (2018). Effect of low-intensity long-duration ultrasound on the symptomatic relief of knee osteoarthritis: a randomized, placebo-controlled double-blind study. *Journal Of Orthopaedic Surgery And Research*.

[11] Nasb M., Huang L. J., Gong C. Z., Hong C. (2020). Human adipose-derived mesenchymal stem cells, low-intensity pulsed ultrasound, or their combination for the treatment of knee osteoarthritis: study protocol for a first-in-man randomized controlled trial. *BMC Musculoskelet Disord*.

[12] Ali K., Dilek B., Sahin Abdulkerim M., Ellidokuz H., Şenocak Ö. (2020). The effectiveness of pulsed ultrasound treatment on pain, function, synovial sac thickness and femoral cartilage thickness in patients with knee osteoarthritis: a randomized, double-blind clinical, controlled study. *Clinical Rehabilitation*.

[13] Rothenberg J. B., Jayaram P., Naqvi U., Gober J., Malanga G. A. (2017). The role of low-intensity pulsed ultrasound on cartilage healing in knee osteoarthritis: a review. *PM R*.

[14] Gul D., Metin Y., Beyazal M. S. (2019). Short-term effects of neuromuscular electrical stimulation and ultrasound therapies on muscle architecture and functional capacity in knee osteoarthritis: a randomized study. *Clinical Rehabilitation*.

[15] Paolillo F. R., Paolillo A. R., Joao J. P. (2018). Ultrasound plus low-level laser therapy for knee osteoarthritis rehabilitation: a randomized, placebo-controlled trial. *Rheumatology International*.

[16] Alfredo P. P., Junior W. S., Casarotto R. A. (2020). Efficacy of continuous and pulsed therapeutic ultrasound combined with exercises for knee osteoarthritis: a randomized controlled trial. *Clinical Rehabilitation*.

[17] Yegin T., Altan L., Aksoy M. K. (2017). The effect of therapeutic ultrasound on pain and physical function in patients with knee osteoarthritis. *Ultrasound in Medicine & Biology*.

[18] Zhang X. G., Sun X. J., Chen G. Q. (2020). Effect of the combinative use of acupotomy therapy and ultrasonic drug penetration in treating knee joint osteoarthritis. *QJM: An International Journal of Medicine*.

[19] Yu W., Zhu S. B., Lv Z. H. (2019). Effects of therapeutic ultrasound for knee osteoarthritis: a systematic review and meta-analysis. *Clinical Rehabilitation*.

[20] Feltham T., Paudel S., Lobao M., Schon L., Zhang Z. (2021). Low-intensity pulsed ultrasound suppresses synovial macrophage infiltration and inflammation in injured knees in rats. *Ultrasound in Medicine & Biology*.

[21] Sangtong K., Chupinijrobkob C., Putthakumnerd W., Kuptniratsaikul V. (2019). Does adding transcutaneous electrical nerve stimulation to therapeutic ultrasound affect pain or function in people with osteoarthritis of the knee? A randomized controlled trial. *Clinical Rehabilitation*.

